RETRACTED

# Application of Visual Sensing Techniques in Computational Intelligence for Risk Assessment of Sports Injuries in Colleges

**DOI:** 10.1155/2022/9080661

**Published:** 2022-04-22

**Authors:** Yan Sun, Yang Zheng, Le He, Liang Guo, Xiao Geng

**Affiliations:** ^1^Department of Physical Education, Chang'an University, Xi'an, Shaanxi 710064, China; ^2^School of Humanity, Chang'an University, Xi'an, Shaanxi 710064, China

## Abstract

Injury prediction is one of the most challenging issues in sports and is a key component of injury prevention, since successful injury prediction forms the basis for effective preventive measures. In this study, an analysis was made on the risk of physical injuries to college students to guarantee the physical safety of students in sports and improve the quality of physical education. Then, a study was carried out on the occurrences of physical injury risks through visual sensing techniques, and an investigation was conducted into the characteristics of physical injury risks in colleges. Next, the student's body shape and physical characteristics are computed using visual sensing techniques, and the risk of sports injuries is evaluated. The results show that the proposed image recognition and computation methods can accurately identify the sports injuries of college students. Furthermore, it can effectively analyze the factors affecting the risk of sports injuries, and the error of the proposed technique remains between −3 and 2. In addition, it can accurately locate the occurrence of sports injury risks and reduce the impact of those risks in time. This work provides technical support for the reduction of sports injury risks and contributes to the improvement of physical education teaching quality in colleges.

## 1. Introduction

Physical education in college has positive effects on health during adolescence. In addition to physical health benefits, physically-active students tend to have better psychological health than their classmates, reporting fewer symptoms of depression, more confidence, self-emotional control, greater social well-being, and higher levels of life satisfaction. Participation in sports also contributes to character development, reducing risk behaviors, improving school performance, and promoting public engagement [1]. Long-term benefits of PE may continue into adulthood, as students who are involved in sports activities may be more likely than their peers to be physically active. However, sports participation may also increase the risk of injuries that cause short-term or long-term disability. Sports injuries are common in younger students. More than 3.4 million teenagers are injured as part of organized sports each year. One-third of all injuries in children are related to sports, too. The most common sports injuries in children are strains and sprains. Contact sports, such as football and basketball, account for more injuries than noncontact sports, such as running and swimming [2].

RETRACTED

To reduce the risk of injuries, the development of college PE is an important link in the development of sports. Presently, college PE is of great significance in enhancing students' physical and psychological health. College PE develops students' confidence and competence to participate in several physical activities that become a dominant part of their lives, both in and out of school [3]. A high-quality PE curriculum enables students to develop different skills and the ability to use strategies and compositional ideas to perform successfully. As a result, they develop the confidence to participate in different physical activities and studies about the value of healthy, active lifestyles. However, because the PE teaching model is different from the traditional teaching methods, there are still many problems in college PE teaching, especially the physical safety of college students in physical education, which needs to be improved [4].

Many scholars have conducted comprehensive research on the assessment of injuries in college physical education. Zhou [5] pointed out that the college PE curriculum plays a very important role in college education, and PE teaching evaluation is the decisive factor for the improvement of physical education. Therefore, to reduce physical injuries and enhance the effects of PE, an important way is to improve the teaching evaluation of college PE. Zadeh et al. [6] predicted that the PE teaching model in the 21st century was still a pattern of coexistence of multiple modes. This diversified pattern was conducive to giving full play to students' subjective initiative, enhancing students' sports awareness, and cultivating students' interest in physical education. Moreover, it will become the main mode of college physical education in China in the 21st century. Zhou [7] revealed that given the problems of physical injuries in the existing college PE program, the way of reform is to change the traditional teaching methods and to realize the sports effect from students' awareness of their physical characteristics. Hulme and Finch [8] found that a combination of high body mass index (BMI) and high mechanical loads could result in injury. Therefore, in creating a physical exercise program, it is essential to incrementally increase mechanical load through the practice season as athletes become conditioned. Rao [9] proposed a dynamic, recursive model for risk assessment and causes of sports injuries and proposed that the injury has a nonlinear behavior. This model is helpful in the understanding of sports injury etiology because it proposes that there may be recurrent changes in susceptibility to injury along with the participation in sports, and the primary risk factors' exposure can produce adaptations and continuously change the risk. Eetvelde [10] has proposed a paradigm shift in sports injuries and emphasized that the literature is limited to consistently identifying predictive factors because current research methods based on unidirectional and logical approaches ignore the factors and complex conditions for sports injury emergence. To reduce sports injuries, Yi and Fang [11] presented a method based on functional motion biological image data and summarized the mistakes and deficits of common movement patterns of athletes and proposed various intervention procedures to improve the effect of sports injury assessment. Jinhai [12] proposed that the machine learning method in combination with image processing can be used to identify athletes at high injury risk during sports participation and to identify risk factors. However, most of the earliest studies did not apply machine learning methods accurately to predict injuries, and the methodological study quality was moderate to very low.

RETRACTED

In this study, a deep perception is implemented on the current situation of college PE. An analysis was made on the risks of sports injuries. Then the potential sports injuries of college students are pointed out to verify the impact of sports injury risks. Furthermore, the college students' body shapes and characteristics of sports injury risks are identified and computed using visual sensing techniques. In addition, an analysis is made on the influencing factors of sports injury risks in colleges, as well as a comprehensive evaluation and technical support is provided for the reforms of college sports education.

The rest of the manuscript is organized as follows: in Section 2, an overview of sports injuries is provided and the proposed visual sensing technique is presented.  Section 3 is about the analysis of the visual sensing techniques. The results are illustrated in Sections 4, and Section 5 is about the conclusion.

## 2. Methods

### 2.1. Sports Injuries in Physical Education

Injuries are common in college sports and have significant physical, psychosocial, and economic consequences. Exploring the injury risk factors and their relationship is thus a crucial component of preventing future injuries in sports [13]. Sports injuries are the results of complex interactions of various risk factors and provoking events making a comprehensive model necessary. Owing to the interactions between extrinsic and intrinsic risk factors as well as their unpredictable nature, the ability to predict the occurrence of an injury event is highly challenging. One of the ultimate tasks in college PE is to prevent the risks that high-intensity physical education will cause to students. These risks refer to the physical and psychological injuries that students may suffer in the process of physical education [14]. This study evaluates the risk of sports injury in colleges through computational intelligence and visual sensing techniques, and reduces the risk through evaluation, to ensure the long-term development of PE in colleges.

RETRACTED

Sports injuries occur during exercise or while participating in a sport. Students are particularly at risk for these types of injuries. Morphological and behavioral characteristics are the most intuitive external manifestations of human body injuries and are important indicators for the evaluation of human health. When predicting human body injuries without contact, the commonly used method is to obtain the image of the human body via infrared-based visual sensing equipment in computational intelligence, and then identify and judge the surface shape of the human body through computation and analysis so that physical safety can be guaranteed for college students in sports. Besides, the risks in the process of PE can be reduced [15].  Figure 1 demonstrates the prediction process of risks to college students in PE through visual sensing techniques in computational intelligence.

Figure 1 reveals that, in the process of physical injury risk assessment for students, what needs to be done initially is to collect information about the physical body shape of students through image acquisition technology. The collected image information is subsequently sent to a processing system. Then, the collected images are processed using different image processing techniques. A comprehensive analysis is conducted on the processed images to evaluate the analyzed images and obtain the results.

### 2.2. Computational Intelligent Vision Sensing Algorithm

When the collected image is input into the computer system, it needs to be processed using visual sensing techniques. After processing, the image can be analyzed and evaluated. In the process of image processing, it is necessary to analyze the gray level of image pixels. Because the equipment in the process of image acquisition has different color recognition mechanisms from human vision, it is necessary to describe the image in terms of RGB (red, green, blue) and HIS (hue, intensity, saturation) color modes in the computer system. The processed image can be more consistent with human visual characteristics. Moreover, the HIS color mode in computer image processing can greatly reduce the task of image processing. The difference between RGB color mode and HIS color mode only lies in the difference in representation methods of the same physical quantity, so they need to be computed and converted. Equations (1)–(3) are the calculations when the light source of the collected image is white [16].

(1) $$\begin{array}{c} H=0.620.170.18=R, \end{array}$$

(2) $$\begin{array}{c} S=00.0661.02=G, \end{array}$$

(3) $$\begin{array}{c} I=0.310.590.11=B, \end{array}$$

where *H* represents the hue, *S* refers to the saturation, and *I* stands for the intensity. The terms *R, G,* and *B* indicate the red, green, and blue, respectively, and · bespeaks the gradient transformation. The calculated image is a gray-level image, which is composed of black and white in human vision. In image analysis, it is also necessary to smooth the collected infrared scanning images to eliminate the image noise, keep the image smooth, reduce the abrupt gradient, and comprehensively improve the image quality [17]. It can be computed as

(4) $$\begin{array}{c} g_{i}=\text{Med}\left(f_{i-v}\ldots f_{i}\ldots f_{i+v}\right)v=\frac{m-1}{2}, \end{array}$$

where *g*_*i*_ represents the filtered value of the image and Med indicates the ordered median. Equation (5) indicates the calculation method for smoothing the two-dimensional image.

(5) $$\begin{array}{c} \;g_{\theta }=\text{Med}\left(x_{ij}\right), \end{array}$$

where *g*_*θ*_ represents the filtered value of a two-dimensional image. Then, in the process of image acquisition, the hierarchical scene of the collected image may be reduced or blurred due to too much brightness or insufficient brightness. Therefore, it is necessary to adjust the contrast of an image to restore the normal visual effect [18], as shown in the following equation:

(6) $$\begin{array}{c} g=T\left(f\right). \end{array}$$

After transformation, the contrast of the processed image can be obtained as

(7) $$\begin{array}{c} g\left(x,y\right)=T\left[f\left(x,y\right)\right], \end{array}$$

where *g*(*x*, *y*) represents the contrast of the processed image and *f*(*x*, *y*) refers to the contrast of the original image. If the contrast of the input image is set as *f*(*x*, *y*) and distributed in [*a*, *b*], the contrast of the output image is *g*(*x*, *y*), distributed in [*m*, *n*], and the relationship between them is linear which can be represented as

(8) $$\begin{array}{c} g\left(x,y\right)=\left\{\begin{array}{cc} m, & f\left(x,y\right)<a,\\ \frac{n-m}{b-a}\left[f\left(x,y\right)-a\right]+m, & a\leq f\left(x,y\right)\leq b,\\ n, & f\left(x,y\right)>b. \end{array}\right. \end{array}$$

The collected image mainly includes the target image of the background. In the analysis process, the target image needs to be extracted; that is, the image is separated to identify the main target image. To achieve this goal, the gray level of the collected image needs to be defined, and the background and target image are separated through the difference in gray value [19], as shown in the following equation:

(9) $$\begin{array}{c} g\left(x,y\right)=\left\{\begin{array}{cc} 1, & f\left(x,y\right)\geq T,\\ 0, & f\left(x,y\right)<T, \end{array}\right. \end{array}$$

where 1 and 0 are the pixel distinction between the background and the target image and  *Tϵ*[*n*_1_, *n*_2_]. The basic principle is to divide the contrast of two images according to the gray value. Assuming that the gray level of an image is 1 ~ *N*, and the pixel of the picture in the gray level *i* is *m*_1_, then the total pixels can be expressed as

(10) $$\begin{array}{c} M=\overset{N}{\underset{i=1}{\sum }}m_{i}. \end{array}$$

The probability calculation accords with equation (11) when the value of gray level is *i*.

(11) $$\begin{array}{c} C_{i}=\frac{m_{i}}{M}. \end{array}$$

In the above equation, *C*_*i*_ represents the obtained probability. If the gray value limit of the image is set to *k*, the pixels of the image can be divided into two gray levels. Equations (12) and (13) signify the calculation process.

(12) $$\begin{array}{c} P_{0}=\left\{1,2,3,\ldots ,k\right\}, \end{array}$$

(13) $$\begin{array}{c} P_{1}=\left\{k+1,k+2,\ldots ,N\right\}. \end{array}$$

Moreover, equation (14) denotes the calculation of the total gray level of the pixels of the image.

(14) $$\begin{array}{c} \beta =\overset{N}{\underset{i=1}{\sum }}C_{i}\cdot i, \end{array}$$

where *P*_0_ and *P*_1_ represent the values of gray levels of the image background and the target image, respectively, and *β* is the total values of gray levels of the image. The average gray level about  *P*_0_ can be computed as

(15) $$\begin{array}{c} \beta_{0}=\overset{k}{\underset{i=1}{\sum }}C_{i}\cdot i. \end{array}$$

Equation (16) demonstrates the pixel calculation under the average gray level.

(16) $$\begin{array}{c} M_{0}=\overset{k}{\underset{i=1}{\sum }}m_{i}. \end{array}$$

The average gray level of *P*_1_ can be computed as

(17) $$\begin{array}{c} \beta_{1}=\beta -\beta_{0}. \end{array}$$

Equation (18) expresses the pixel calculation under the average gray level.

(18) $$\begin{array}{c} M_{1}=M-M_{0}. \end{array}$$

Equations (19) and (20) compute the ratio between the background and the target image

(19) $$\begin{array}{c} \rho_{0}=\overset{k}{\underset{i=1}{\sum }}C_{i}=\rho \left(k\right), \end{array}$$

(20) $$\begin{array}{c} \rho_{1}=1-\rho \left(k\right). \end{array}$$

The processing on *P*_0_ and *P*_1_ can be computed using equations (21) and (22), respectively.

(21) $$\begin{array}{c} \beta_{0}=\frac{\beta \left(v\right)}{\rho \left(k\right)}, \end{array}$$

(22) $$\begin{array}{c} \beta_{1}=\frac{\left[\beta -\beta \left(k\right)\right]}{\left[\beta -\beta \left(k\right)\right]}. \end{array}$$

The computation of the total average value of the processed image is as follows:

(23) $$\begin{array}{c} \beta =\rho_{0}\beta_{0}+\rho_{1}\beta_{1}. \end{array}$$

Equation (24) computes the variance between species *P*_0_ and *P*_1_.

(24) $$\begin{array}{c} \sigma^{2}\left(k\right)=\rho_{0}{\left(\beta -\beta_{0}\right)}^{2}+\rho_{1}{\left(\beta -\beta_{1}\right)}^{2}=\rho_{0}\rho_{1}{\left(\beta_{0}-\beta_{1}\right)}^{2}. \end{array}$$

The processed image is the best object for analysis. After analysis, the risks in the process of college students' physical education can be evaluated to guarantee their physical safety [19].

RETRACTED

## 3. Analysis of Factors Causing Sports Injuries

With the increase of people's exercise in today's society, how to exercise scientifically and healthily has attracted much attention. Therefore, sports injury risk assessment and monitoring systems have attracted more and more attention in terms of real-time, flexibility, intelligence, and other aspects. It is indispensable to conduct a risk assessment in the process of implementing high-intensity physical education in colleges. To explore the sports injury assessment process, it is essential to identify the factors that may cause sports injuries to college students during sports activities [20].

The identification of the causes of injury is an important step in injury prevention as this can be used to develop active injury prevention programs. Sports professionals need to know why some athletes may be at risk of injury risk factors and how injuries occur to understand the causes of sports injuries. Sports injuries are rarely due to a single factor, and can generally be attributed to an association of circumstances [21]. These injury risk factors can be categorized into extrinsic and intrinsic injury risk. The extrinsic risk factor mainly includes human factors (e.g. opponents, teammates), sports factors (e.g. rules, referees, coaching), and environmental factors such as weather, ice conditions, floor and turf type, and playing surface. The internal risk factors mainly include age, sex, body composition, skill level, psychological factors, and physical fitness. Interaction between the extrinsic and intrinsic risk factors may cause a student to be more or less prone to injury. A combination of external and internal risk factors acting concurrently puts students at a higher risk for injury [22].  Figure 2 lists the factors that may cause sports injuries to students in the process of obtaining a college sports education.

RETRACTED

This study first recognizes the influencing factors, then analyzes the injury status of students according to the impact of different factors based on the occurrence of risk status, and finally formulates corresponding guidelines for college sports education according to the results to guarantee students' physical safety in sports [23].

Figure 3 displays the specific process of risk identification. This implies that, in the identification of sports injury risk, first, it is necessary to monitor the physical characteristics of students participating in sports to confirm whether they have sports injuries. If not, other students need to be monitored. If yes, the causes of sports injuries in students are analyzed and certain rules are formulated according to the causes of injuries to prevent the recurrence of such sports injuries again [22, 23]. In this study, two groups of students, 30 in each group, were monitored for sports injuries through visual sensing techniques, and 30 students with sports injuries were selected to analyze the factors of injuries. Finally, relevant suggestions were put forward according to the results.

## 4. Comprehensive Analysis

### 4.1. Detection of Students' Sports Injuries

Sports injuries are a composite emergent phenomenon. Using visual sensing techniques, the sports injuries of college students can be evaluated. It can be used to accurately check whether students have sports injuries, to effectively guarantee students' physical and mental health, and to comprehensively improve the quality of physical education teaching in colleges.  Figure 4 manifests the proportion of sports injuries suffered by college students.

It can be seen that, by checking whether 30 people in each group have sports injuries and checking their body shape and physical characteristics through visual sensing techniques, different degrees of sports injuries are found in each sports event. Among them, the number of sports injuries in ball games is the largest in terms of the number of the two groups. A total of 28 students have suffered sports injuries of varying degrees in ball games. A total of 35 students have suffered sports injuries of varying degrees in the horizontal bar. The number of sports injuries from the long jump and high jump is the least, and the total number is 11. It implies that the evaluation of sports injuries of college students is necessary. Through an analysis of sports injuries, the problems faced by most students in sports can be detected.  Figure 5 signifies the comparison between the actual results and the results in the students' sports injury detection.

RETRACTED

Figure 5 reveals that, in the comparison between the detected results and the actual results of the two groups, the error in the detected results of group 1 is about ±2, and the detected results of two movements are completely consistent with the actual results. The error in the detected results of group 2 is about ±3, of which there is one movement, and the detected results are completely consistent with the actual results. Hence, by analyzing the images of students' body shapes and characteristics through visual sensing techniques, the students' having sports injuries can be effectively verified.

### 4.2. Analysis of Factors Involved in Sports Injuries

Further analysis of the factors of sports injuries reveals that the detected results are consistent with the actual results, which can be used to put forward constructive normative opinions on college students' sports education, improve students' comprehensive quality in sports, and provide guidelines for the improvement of sports education quality.  Figure 6 manifests the self-factors of sports injuries in the two groups of students.

Figure 6 reveals that, among the self-factors (intrinsic factors) S (skill), PF (physical fitness), OI (old injuries), MQ (mental quality), and MS (mental state) of sports injuries in students, physical fitness has the greatest impact on sports injuries. In the test results, the numbers of sports injuries caused by the poor physical fitness of members were 5 and 6 in the two groups, respectively. The factor with the lowest comprehensive impact is the mental state of students. In the test results, the numbers of sports injuries caused by mental state were 1 and 0 in the two groups, respectively. Physical quality is very important in sports, and psychological factors will also have a certain impact. Therefore, college physical education needs to be comprehensively improved.  Figure 7 displays the external (extrinsic factors) factors of sports injury in the two groups of students.

Figure 7 indicates that, among the external factors *T* (time), W (weather), S (site), *M* (management), and A (attitude) of sports injuries in the two groups, the weather is the most influential factor. In the test results, the number of sports injuries caused by weather is 12 and 13 in the two groups, respectively, and the lowest comprehensive impression factor is the students' attitude to the outside world. In the test results, the numbers of sports injuries due to external attitudes were 4 and 2, respectively in the two groups. More attention needs to be paid to the weather conditions in the process of sports so that college physical education can also be carried out scientifically. In the prediction of the external environment, the image analysis of students' body shapes and characteristics is carried out by using visual sensing techniques, and there are ideal results of the comparison between the obtained results and the actual results.  Figure 8 displays the errors in sports injuries detection of college students.

RETRACTED

Figure 8 indicates that, in the analysis of the error factors in sports injuries, the detection error of self-factors is about ± 2, while the detection error of external factors is between −3 and 2. It is close to the results of the sports injuries obtained by analyzing the characteristics of students' body shapes through the visual sensing technique and the actual sports injuries.

The study analyzed the body shape and characteristics of college students using visual sensing, image recognition, and image processing techniques. The purpose is to detect college students' sports injuries and analyze the influencing factors. It comprehensively evaluates the risk of college sports injuries through detection and analysis. It is found that sports injuries in colleges occur in various sports events. It is essential to improve the existing sports teaching mode, reduce the risk of sports injuries in sports education, and guarantee students with safety in sports education. Among students' self-factors, colleges should focus on basic physical education, enhance students' physical fitness and sports skills training, and also provide psychological counseling and education for students. Then, college administration should also cooperate with parents to vigorously support students' sports training, build good sports venues, manage students' sports education, and provide proper time for sports. These aspects can provide a basic guarantee for preventing sports injuries in college sports education.

## 5. Conclusion

Injuries are common in college sports and can have significant physical, psychosocial, and financial consequences. Identification of sports injury risk factors and their relationship is, therefore, a key component in reducing future injuries in sports. In this study, an analysis was made on the risk of physical injuries to college students to guarantee the physical safety of students in sports and improve the quality of physical education. Then, a study is carried out on the occurrence of physical injury risk through visual sensing techniques, and an investigation is made into the characteristics of physical injury risk in colleges. It is found that among the intrinsic sports risk factors, physical fitness has the greatest impact on sports injuries, whereas in the case of extrinsic factors, unfavorable weather is the main cause of sports injuries. Finally, by comparing the detected results with the actual results, it is concluded that the image recognition and processing techniques can accurately identify the occurrence of sports injuries in college students and can effectively identify the factors that cause sports injuries. The present work provides technical support for the detection of sports injuries in colleges and contributes to the improvement of sports education quality in colleges.

RETRACTED

## Figures and Tables

**Figure 1:** Risk assessment of physical education students by visual sensing techniques.

**Figure 2:** Factors causing sports injury in colleges.

**Figure 3:** Risk identification of sports injuries.

**Figure 4:** Sports injury detection of College Students.

**Figure 5:** Comparison between actual sports injuries and detected sports injuries: (a) the comparison between actual sports injuries and detected sports injuries in group 1 and (b) the comparison between actual sports injuries and detected sports injuries in group 2.

**Figure 6:** Self-factors of sports injury in colleges: (a) the self-factors of group 1 and (b) the self-factors of group 2.

**Figure 7:** External factors of sports injury in colleges: (a) group 1 and (b) group 2.

**Figure 8:** The number of error factors in sports injuries of college students: (a) self-factors and (b) external factors.

## Data Availability

The data used to support the findings of this study are available from the corresponding author upon request.

## References

[1] Xin C., Wang X. (2020). Research on the application of college physical education teaching mode in the cloud computing environment. *Journal of Physics: Conference Series*.

[2] Shi X., Li X., Wu Y. (2021). The Application of computer-aided teaching and mobile Internet terminal in college physical education. *Computer-Aided Design*.

[3] Kim H., Song T., Lim S., Kohl H. W., Han H. (2021). Physical activity engagement outside of college physical education: application of the transtheoretical model. *American Journal of Health Behavior*.

[4] Yu S. A. (2021). Application of computer information technology in college physical education using fuzzy evaluation theory. *Computational Intelligence*.

[5] Zhou H. (2021). Research on the Function of Computer Aided Teaching in College Physical Education. *Conference Series*.

[6] Zadeh A., Taylor D., Bertsos M., Tillman T., Nosoudi N., Bruce S. (2020). Predicting Sports Injuries with Wearable Technology and Data Analysis. *Information Systems Frontiers*.

RETRACTED

[7] Meeuwisse W. H., Tyreman H., Hagel B., Emery C. (2007). A dynamic model of etiology in sport injury: the recursive nature of risk and causation. *Clinical Journal of Sport Medicine*.

[8] Hulme A., Finch C. F. (2015). From monocausality to system thinking: a complementary and alternative conceptual approach for better understanding the development and prevention of sports injury. *Inj Epidemiol*.

[9] Rao F. (2021). Experimental study on alleviating sports injury through data screening of functional motor biological images. *Journal of Healthcare Engineering*.

[10] Eetvelde H. V., Mendonca L. D., Ley C., Seil R., Tischer T. (2021). Machine learning methods in sports injury prediction and prevention: a systematic review. *Journal of Experimental Orthopedics*.

[11] Yi W., Fang F. (2019). The design and realization of the management system of college physical education under the network environment. *Journal of Physics: Conference Series*.

[12] Jinhai Y. (2019). Research on the application of big data ecology in college physical education and training. *IOP Conference Series: Materials Science and Engineering*.

[13] Vaughn M., Hur J. W., Russell J. (2019). Flipping a college physical activity course: impact on knowledge, skills, and physical activity. *Journal of Pedagogical Research*.

[14] Feng C. (2020). Research on the application of computer virtual reality technology in college physical education teaching. *Journal of Physics: Conference Series*.

[15] Deng C., Tang Z., Li X., Zhao Z. (2020). Construction and application of web-based resource repository of college physical education. *Journal of Physics: Conference Series*.

[16] Lei P. (2021). Research on the quality of online teaching of college physical education courses under the impact of the epidemic. *Journal of Frontiers in Educational Research*.

[17] Li J. (2020). Application research of vision sensor in material sorting automation control system. *IOP Conference Series: Materials Science and Engineering*.

[18] Xiao R., Xu Y., Hou Z., Chen C., Chen S. (2019). An adaptive feature extraction algorithm for multiple typical seam tracking based on vision sensor in robotic arc welding. *Sensors and Actuators A: Physical*.

[19] Fan J., Jing F., Yang L., Long T., Tan M. (2019). A precise seam tracking method for narrow butt seams based on structured light vision sensor. *Optics & Laser Technology*.

[20] Han Y., Fan J., Yang X. (2020). A structured light vision sensor for on-line weld bead measurement and weld quality inspection. *International Journal of Advanced Manufacturing Technology*.

RETRACTED

[21] Du J., Xie D., Zhang Q. (2021). A robust neuromorphic vision sensor with optical control of ferroelectric switching. *Nano Energy*.

[22] Bhowmik P., Pantho M. J. H., Bobda C. (2021). Bio-inspired smart vision sensor: toward a reconfigurable hardware modeling of the hierarchical processing in the brain. *Journal of Real-Time Image Processing*.

[23] Oudah M., Al Naji A., Chahl J. (2020). Hand gesture recognition based on computer vision: a review of techniques. *Journal of Imaging*.

